RETRACTED

# Female Colon Cancer Metastasis Pattern and Prognosis: A SEER-Based Study

**DOI:** 10.1155/2022/3865601

**Published:** 2022-07-07

**Authors:** Yurong Liu, Rongbin Kang, Huida Zheng, Pengcheng Wang, Weixin Jiang, Bin Xiong, Jintao Chen, Jianhua Xu

**Affiliations:** ^1^Department of Gastrointestinal Surgery, The Second Affiliated Hospital of Fujian Medical University, Quanzhou, China; ^2^Department of Gastric Surgery, Fujian Medical University Union Hospital, Fuzhou, China; ^3^Department of Endocrinology, The Affiliated Hospital of Qingdao University, Qingdao, China

## Abstract

The purpose of this study was to compare the metastatic pattern and prognosis of female colon cancer (FCC) to that of male colon cancer (MCC) to ascertain the independent factors impacting the prognosis of patients with FCC. The data of the present study population were retrieved from the Surveillance, Epidemiology, and End Results (SEER) database. Descriptive analysis, the Kaplan-Meier method, and the Cox regression were used to evaluated FCC characteristics and factors associated with prognosis. There were 56,442 patients diagnosed with FCC, of whom 8,817 had distant metastases. Compared to patients with nonmetastatic FCC, a greater proportion of metastatic FCC patients was less than 60 years of age, black race, and grade III-IV. The primary sites were mainly located on the left side and have more possibility to receive chemotherapy and radiotherapy. Compared to metastatic MCC, a higher proportion of metastatic FCC patients ranged over 60 years of age, black race, treated without chemotherapy, and insurance, while the primary site was located on the right side. Liver and lung were the two most common sites of solitary metastases in CC, and among patients with solitary metastases in CC, patients who had lung metastases had a better prognosis than those who developed other types of metastasizes. Patients with FCC with metastases of the liver had a worse prognosis than their MCC counterparts. Cox multivariate regression analysis showed that the risk ratio was higher in metastatic FCC patients compared to those without metastases. We report the survival comparison of metastatic FCC with nonmetastatic FCC through the SEER database. Our results suggest that it has unique clinicopathological features and differs from metastatic MCC. Furthermore, patients with liver metastatic FCC have a worse prognosis than those with MCC. Emphasis on screening for colon cancer in women and additional clinical care should be paid for, especially for patients with FCC with metastatic liver cancer.

## 1. Introduction

Colon cancer (CC) is the third most prevalent cancer in the United States, occurring in both men and women, and is also the third leading cause of mortality from cancer [1]. The cumulative risk of developing colon cancer before 75 years is 1.51% and 1.12% for men and women, respectively, giving a rate of 1 in 66 men and 1 in 89 women to develop CC [2]. Despite recent advances in chemotherapy and radiotherapy for CC, surgical resection remains the primary treatment, but there are gender differences in CC treatment choices [3, 4].

RETRACTED

In general, gender may be the first patient characteristic to be considered when discussing tumor differences between patient subgroups. Gender differences in tumor behavior exist in patients with colon cancer [5], but the exact mechanisms are unknown. The high mortality rate of colon cancer is mainly due to distant metastases, and the degree of CC differentiation and histopathological type is all factors that affect the prognosis of CC patients [6, 7], while the clinical characteristics, metastatic patterns, and factors related to the prognosis in FCC with distant metastases have not been thoroughly described, which means these variables in the patient populations remain in uncharted territory for this type of disease to be explored. Thus, we identified the FCC data recorded in this study from 2010 to 2015 in the SEER database. We conducted cross-sectional and longitudinal studies of patients with metastatic FCC to determine their clinicopathological characteristics and differences from patients with metastatic MCC and identify independent factors that affect the prognosis of patients with FCC.

## 2. Method

### 2.1. Populations and Characteristics

The data for this study were extracted from the National Cancer Institute's SEER-18 database, using the National Cancer Institute's SEER^∗^Stat version 8.3.9 (http://http://www.seer.cancer.gov/seerstat). Patients included in the study were those ≥18 years old histologically diagnosed with colon cancer between 2010 and 2015. The inclusion criteria were as follows: (a) ICD-O-3 site codes: cecum, ascending colon, hepatic flexure of colon, transverse colon, splentic flexure of colon, descending colon, and sigmoid colon; overlapping lesion of colon and colon NOS; (b) colon cancer was the only primary malignancy; and (c) patients who were under active follow-up; furthermore, patients who met the following criteria were excluded: (a) patients with additional primary cancers, (b) patients with no information on the status of distant organ metastases, (c) unknown autopsy or death certificate diagnoses and diagnoses not confirmed by pathology, and (d) unknown survival months. After completing the necessary screening, we were able to identify 114039 individuals who were qualified for survival analysis and other investigations (Figure 1).

RETRACTED

The patients were separated into two groups: FCC and MCC. The AJCC 7th edition was used to determine clinicopathological staging [8]. Age, race, primary site, histology, pathological grade, AJCC TNM stage, surgery, radiotherapy and chemotherapy information, marital status, and insurance status were included as research parameters.

### 2.2. Statistical Analysis

To summarize demographic and clinical factors, we performed descriptive statistics. The Pearson chi-square test and Fisher exact probability method were utilized to evaluate clinicopathological variables between cohorts. The overall survival (OS) of patients with MCC and FCC with distinct metastatic organs was analyzed by Kaplan-Meier and log-rank test. In addition, we looked for other factors that could impact prognosis using univariate and multivariate Cox proportional risk models. All the tests were two-sided, and statistical significance was defined as *P* < 0.05. The SEER^∗^Stat program version 8.3.9 was used to collect all of the data. All statistical analyses were conducted using *R* software version 4.0.4.

## 3. Results

### 3.1. Patient Clinicopathological Data

A total number of 56442 FCC patients were enrolled in the study. 8817 cases (15.6%) of these FCC patients had distant metastases. A higher proportion of FCC patients with distant metastases were younger than 60 years, black, grades III-IV receiving chemotherapy and radiotherapy, and married than FCC patients without metastases. The proportion of patients with the primary site in the right colon, surgery, and insurance was lower.  Table 1 shows the detailed patient clinical characteristics. Patients with FCC with distant organ metastases had more diagnoses than MCC age > 60 years, black race, right colon, unmarried, and with insurance; the former were less likely to receive chemotherapy than the latter. Both groups had identical pathology, pathological grading, TN stage, surgery, and radiation.

FCC: female colon cancer; MCC: male colon cancer. ^Comparison between male colon cancer without metastasis and male colon cancer with metastasis. ^∗^Comparison between male colon cancer with metastasis and female colon cancer with metastasis. ^#^Comparison between female colon cancer without metastasis and female colon cancer with metastasis. ^∗^*P* < .05, ^∗∗^*P* < .001.

### 3.2. Metastasis Pattern

The majority (76.56%) of the cohort of FCC with distant metastasis had single site distant metastases. The most common location of metastases was the liver, which represented 68.49% of the patients. The number of lung metastasis accounted for 593 (6.73%). Very few patients had bone or brain metastasis. Concerning the differences in metastasis patterns between FCC and MCC, MCC patients had a lower proportion of brain metastases only than their FCC counterparts (0.33% vs 0.53%), as well as lung metastases only (5.5% vs 6.73%), whereas the percentage of bone and liver metastases was higher in MCC patients (Table 2).

RETRACTED

### 3.3. Survival Analysis

Among patients with metastatic colon cancer by gender, liver metastases only, lung metastases only, and combined liver metastases with lung metastases accounted for more than 90% of the total metastatic population. We included these three groups in our survival and prognosis analyses to investigate the influence of distant metastases on prognosis. Kaplan-Meier analysis showed that for patients with liver metastases only, the survival rate of MCC patients was better than that of FCC patients and was statistically significant (*P* = 0.0058), while for the other two groups, our analysis showed no statistical difference in OS by gender (Figure 2).

However, it appears that patients between those three groups and nonmetastatic FCC were significantly different (Figure 3).

Survival rates decreased as the number of metastatic sites increased in patients with metastatic FCC (Figure 4).

The Cox univariate analysis revealed that age, race, tumor primary site, histopathology type, pathology grade, TN stage, surgery, chemotherapy, marital status, insurance situation, and the metastatic sites were independent factors affecting OS (*P* < 0.001), and these variables were included in the multivariate model (Table 3). In detail, black, age > 60 years, primary tumor site in the right colon or the overlapping lesion, nonadenocarcinoma, pathological grade II, grade III, and grade IV, distant metastasis, treatment without surgery and chemotherapy, single, and distant metastasis correlated with poor prognosis. Radiation therapy did not affect the outcome of this study.

## 4. Discussion

In both men and women, colon cancer is one of the most prevalent causes of cancer development. Despite recent advances in CC screening, diagnosis, and treatment, the long-term prognosis of CC patients remains poor [8]. The prognosis of patients with metastatic and nonmetastatic FCC was compared with patients with MCC. To our knowledge, this study is the first gender-focused metastasis model-based analysis of colon cancer data.

In this study, the metastasis rate was 17.9% versus 15.6% in male versus female colon cancer patients, respectively. The incidence of colon cancer increased significantly with age. According to past research, younger CC patients are more likely to develop metastases than older patients and have limited surgical and chemotherapeutic treatment [9]. Similarly, younger CC patients in this study developed metastases significantly more than older CC patients, and when women were diagnosed with colon cancer, they were significantly older than men and presented with more severe disease. This may be explained by the lower rate of screening colonoscopy in women over 65 years of age than men of the same age [10]. A higher rate of incomplete colonoscopy in women has also been reported [11], contributing to more colon cancers in women of advanced age. The population was more than 3/4 white in the data we included, but we found that black CC patients were more likely to have distant metastases, consistent with previously reported results [12]. Previous studies have demonstrated a lack of awareness of screening guidelines in general and in African American men in particular [13, 14].

RETRACTED

Furthermore, black patients with metastatic colorectal cancer are less likely to get chemotherapy or have liver metastasectomy, and they are less likely to discuss or contemplate participating in studies [15, 16]. The primary location of the tumor is strongly associated with patient prognosis, as reported in different types of cancer [17–19]. In the same vein, Ishihara et al. [20] found that proximal indolent cell carcinoma is considered a distinct subgroup with a good tumor prognosis in colon cancer. Our analysis from a gender perspective showed that the primary tumor location of FCC was more often located in the right colon than MCC, which is consistent with previous reports [4]. In patients with colon cancer, researchers developed a nomogram that predicted risk variables for liver and lung metastasis, with tumor site being an independent risk factor for metastasis [21]. As we mentioned earlier, women have a higher rate of incomplete colonoscopy [9]. In addition, some women tend to have a more extended colon cross-section and smaller bowel diameter, making standard colonoscopy equipment usually unsuitable for this group of women [22]. Therefore, we recommend that women need to choose a thinner colonoscopy device for a complete colonoscopy when undergoing colon cancer screening to reduce the number of missed right colon cancer due to the device and physiological configuration.

The preference for chemotherapy and radiation therapy over surgery in advanced cancers may also explain why patients with metastatic FCC rarely undergo surgery. However, treatment of stage IV colon cancer remains challenging, and despite recent advances in chemotherapy and other palliative treatment modalities, the best treatment options for colon cancer with unresectable metastases remain to be elucidated. Interestingly, the number of patients treated with radiation is more than 6% for male and female patients. Adjuvant external beam radiation is usually not recommended due to the difficulty of targeting and the proximity of critical surrounding structures (e.g., small intestine), as these factors can limit the dose that can kill the tumor. Recent findings show that adjuvant radiotherapy can significantly prolong OS in patients with advanced local disease (pT4) and positive cut margins [23]; therefore, adjuvant therapy for CC patients should not be abandoned due to the limitations of RT. Hypodifferentiated versus undifferentiated colon cancer is more likely to develop distant metastases, and there is no difference between men and women.

RETRACTED

Although modern research has been able to elucidate the pathogenesis of CC and provide effective screening strategies, the prevalence of CC is still increasing. A better understanding of the occurrence, progression, and metastasis of CC can help develop molecular markers for early detection and risk stratification methods to improve clinical care for CC patients. We compared distant metastasis patterns in patients with MCC and FCC in depth using the SEER database to understand the survival differences between patients with different metastasis patterns. Single-site metastases occurred in more than three-quarters of the total number of patients. Overall, the liver and brain were the most common and least common sites of solitary metastases in patients with CC, respectively, consistent with prior reports [24]. Due to the blood-brain barrier, fewer patients had brain metastases alone (0.33% vs. 0.53%), but when combined with metastases from other sites, brain metastases exceeded 1% in both sexes.

Similarly, when lung metastases were combined with liver metastases, the number of patients was much higher than that of patients with lung metastases alone. We believe that once a tumor develops distant metastasis in one organ, it may accelerate metastasis in other sites; although, brain metastasis alone is uncommon when it has metastasis in other sites. Interestingly, FCC was more likely to have a single lung metastasis than MCC; yet, we found no significant difference in their OS.

The clinicopathological characteristics and metastatic patterns of metastatic MCC and FCC were different in the present study. Multivariate Cox regression showed that in patients with FCC, advanced age, primary site in the right colon, higher pathological grade, and distant organ metastasis were independent risk factors affecting the prognosis of patients with FCC (Table 3). The most common site of distant metastasis in patients with CC is the liver, but we found differences in prognosis by gender, and the survival of patients with single liver metastasis in FCC was significantly lower than that of MCC in the same group (*P* = 0.0058). Once the tumor metastasized, patient survival decreased, the OS decreased more with increasing metastatic sites, and the same results have been reported in other tumors [24, 25]. Liver and lung are the two most common sites of solitary metastases in FCC [26], but there are differences in OS in patients with these two metastases. The OS of patients with solitary lung metastasis was significantly higher than that of patients with solitary liver metastasis. Reasons for the difference still need further exploration. However, there are some limitations which worth further more research in this study; firstly, the BMI and BSA of patients were not included in this study, and the prospective study already completed by Thygesen et al. [27] demonstrated that obesity and overweight are key variable risk factors for colon cancer. With this finding, they advocate public health interventions to avoid risks due to weight gain as a way to better prevent colon cancer. Secondly, the data source used in this study was the SEER database. We were only able to study this with the available information on four organ metastases, namely, liver, lung, bone, and brain, due to the inability to obtain data on other metastasis sites, and we cannot conduct a more comprehensive study. Finally, there are differences in metastatic patterns between males and females, but we could not determine which factors are associated with them. That said, further research to clarify the rationale underlying these differences is necessary.

RETRACTED

## 5. Conclusion

Our population-based analysis of 114,039 CC patients found that older women were diagnosed with colon cancer, and that advanced age at diagnosis (>60 years) significantly predicted worsening OS. The primary site of FCC was more likely to be in the right colon. Female patients may be more likely to have pulmonary metastases; although the most common distant sites of metastasis for both FCC and MCC are liver and lung, patients with liver metastases from FCC have a worse prognosis than their MCC counterparts, and we also found that patients with liver metastases from FCC have a worse prognosis than those with pulmonary metastases. The results of this study have some reference value for clinicians in dealing with CC patients, who should pay attention to colon cancer screening in women and should actively receive treatment for FCC patients with liver metastases and lung metastases to improve their prognosis.

## Figures and Tables

**Figure 1:** Flowchart of selection of patients with metastatic colon cancer used the SEER database. SEER: surveillance epidemiology and end results.

RETRACTED

**Figure 2:** OS rate of MCC and FCC patients at different metastasis sites. (a) OS of liver alone metastasis between MCC and FCC patients. (b) OS of lung alone metastasis between MCC and FCC patients. (c) OS of both liver and lung metastasis between MCC and FCC patients. FCC: female colon cancer; MCC: male colon cancer; OS: overall survival.

**Figure 3:** The survival difference among the different metastasis sites in FCC patients. FCC: female colon cancer.

**Figure 4:** The survival difference among the different numbers of metastasis sites in FCC patients. FCC: female colon cancer.

**Table 1:** Clinical characteristics of male and female patients with colon cancer.

	MCC without metastasis		MCC with metastasis		FCC without metastasis		FCC with metastasis		*P* value^	*P* value^∗^	*P* value^#^
	*N* = 47277	% 82.1	*N* = 10320	% 17.9	*N* = 47625	% 84.4	*N* = 8817	%15.6			
Age at diagnosis (year)									.000^∗∗^	.000^∗∗^	.000^∗∗^
≤60	17668	37.4	4430	42.9	14952	31.4	3546	40.2			
>60	29609	62.6	5890	57.1	32673	68.6	5271	59.8			
Race									.000^∗∗^	.000^∗∗^	.000^∗∗^
Black	5541	11.7	1652	16.0	6292	13.2	1617	18.3			
White	36598	77.4	7727	74.9	36343	76.3	6362	72.2			
Others	4570	9.67	919	8.91	4522	9.50	822	9.32			
Unknown	568	1.20	22	0.21	468	0.98	16	0.18			
Primary site									.000^∗∗^	.000^∗∗^	.000^∗∗^
Right colon	22445	47.5	4243	41.1	26482	55.6	4183	47.4			
Left colon	23686	50.1	5264	51.0	20023	42.0	3812	43.2			
Overlapping lesion	532	1.13	138	1.34	570	1.20	132	1.50			
Unknown	614	1.30	675	6.54	550	1.15	690	7.83			
Histopathology type									.000^∗∗^	0.912	.000^∗∗^
Adenocarcinoma	45618	96.5	9742	94.4	45729	96.0	8319	94.4			
Others	1659	3.51	578	5.60	1896	3.98	498	5.65			
Pathology grade									.000^∗∗^	0.063	.000^∗∗^
(I) Well-differentiated	4399	9.30	382	3.70	4197	8.81	333	3.78			
(II) Moderately	30045	63.6	5326	51.6	29583	62.1	4390	49.8			
(III) Poorly differentiated	5895	12.5	1841	17.8	7334	15.4	1577	17.9			
(IV) Undifferentiated	1244	2.63	348	3.37	1615	3.39	337	3.82			
Unknown	5694	12.0	2423	23.5	4896	10.3	2180	24.7			
T									0.000	0.697	0.000
T0-T2	18260	38.6	1276	33.9	17413	36.6	1055	12.0			
T3-T4	27645	58.5	6175	59.8	28741	60.3	5293	60.0			
Unknown	1372	2.9	2869	27.8	1471	3.1	2469	28.0			
N									0.000	0.117	0.000
N0	30765	65.1	3199	31.0	30468	64.0	2786	31.6			
N1	10342	21.9	3382	32.8	10681	22.4	2746	31.1			
N2	5501	11.6	2520	24.4	5788	12.2	2222	25.2			
Unknown	699	1.4	1219	11.8	688	1.4	1063	12.1			
Surgery									.000^∗∗^	0.356	.000^∗∗^
No	2635	5.57	4653	45.1	2625	5.51	3958	44.9			
Yes	44578	94.3	5647	54.7	44939	94.4	4849	55.0			
Unknown	64	0.14	20	0.19	61	0.13	10	0.11			
Radiotherapy									.000^∗∗^	0.145	.000^∗∗^
No	45314	95.8	9715	94.1	46271	97.2	8344	94.6			
Yes	1963	4.15	605	5.86	1354	2.84	473	5.36			
Chemotherapy									.000^∗∗^	.000^∗∗^	.000^∗∗^
No	33412	70.7	3473	33.7	34496	72.4	3227	36.6			
Yes	13865	29.3	6847	66.3	13129	27.6	5590	63.4			
Marital status									.000^∗∗^	.000^∗∗^	.000^∗∗^
Married	28733	60.8	5875	56.9	20114	42.2	3757	42.6			
Unmarried	15497	32.8	3931	38.1	24252	50.9	4600	52.2			
Unknown	3047	6.44	514	4.98	3259	6.84	460	5.22			
Insurance situation									.000^∗∗^	0.011^∗^	.000^∗∗^
Insurance	44271	93.6	9549	92.5	45093	94.7	8254	93.6			
No insurance	1658	3.51	585	5.67	1286	2.70	419	4.75			
Unknown	1348	2.85	186	1.80	1246	2.62	144	1.63			

FCC: female colon cancer; MCC: male colon cancer. ^Comparison between male colon cancer without metastasis and male colon cancer with metastasis. ^∗^Comparison between male colon cancer with metastasis and female colon cancer with metastasis. ^#^Comparison between female colon cancer without metastasis and female colon cancer with metastasis. ^∗^*P* < .05; ^∗∗^*P* < .001.

RETRACTED

**Table 2:** Comparison of organ metastasis patterns between male and female patients with colon cancer.

Variable	Male		Female		*P* value
	*N* = 10320		*N* = 8817		
	*n*	%	*n*	%	
Bone metastasis only	100	0.97	71	0.81	0.230^∗^
Brain metastasis only	34	0.33	47	0.53	0.031^∗^
Liver metastasis only	7107	68.87	6039	68.49	0.579^∗^
Lung metastasis only	568	5.50	593	6.73	<.001^∗^
Bone and brain	4	0.04	4	0.05	0.824^∗^
Bone and liver	275	2.66	196	2.22	0.049^∗^
Bone and lung	52	0.50	40	0.45	0.617^∗^
Brain and liver	29	0.28	23	0.26	0.790^∗^
Brain and lung	22	0.21	17	0.19	0.756^∗^
Liver and lung	1826	17.69	1564	17.74	0.936^∗^
Bone, brain, and liver	11	0.11	8	0.09	0.729^∗^
Bone, brain, and lung	6	0.06	4	0.05	0.700^∗^
Bone, liver, and lung	222	2.15	165	1.87	0.171^∗^
Brain, liver, and lung	40	0.39	36	0.41	0.820^∗^
Bone, brain, liver, and lung	24	0.23	10	0.11	0.051^∗^
One site metastasis	7809	75.67	6750	76.56	0.151^∗^
Two site metastasis	2208	21.40	1844	20.99	0.498^∗^
Three site metastasis	279	2.70	213	2.42	0.210^∗^
Four site metastasis	24	0.23	10	0.11	0.051^∗^

^∗^Pearson chi-squared test.

**Table 3:** Univariate and multivariate survival analysis of female colon cancer patients with liver alone, lung alone, and simultaneous liver and lung metastasis.

Characteristics	Univariate analysis	Multivariate analysis		
	*P* value	Hazard ratio	95% CI	*P* value
Age at diagnosis (year)	<.001			<.001
≤60		Reference		
>60		1.78	1.72-1.84	<.001
Race	<.001			<.001
Black		Reference		
White		0.98	0.95-1.02	0.4443
Others		0.84	0.79-0.90	<.001
Unknown		0.11	0.07-0.19	<.001
Primary site	<.001			<.001
Right colon		Reference		
Left colon		0.87	0.84-0.90	<.001
Overlapping lesion		1.15	1.03-1.28	0.0154
Unknown		1.27	1.18-1.39	<.001
Histopathology type	<.001			<.001
Adenocarcinoma		Reference		
Others		1.17	1.1-1.24	<.001
Pathology grade	<.001			<.001
(I) Well-differentiated		Reference		
(II) Moderately		1.15	1.08-1.23	<.001
(III) Poorly differentiated		1.62	1.51-1.74	<.001
(IV) Undifferentiated		1.94	1.77-2.11	<.001
Unknown		1.17	1.09-1.26	<.001
T stage	<.001			
T0-T2		Reference		
T3-T4		1.93	1.85-2.01	<.001
Unknown		1.53	1.44-1.63	<.001
N stage	<.001			
N0		Reference		
N1		1.70	1.63-1.76	<.001
N2		3.22	3.09-3.37	<.001
Unknown		1.32	1.23-1.41	<.001
Surgery	<.001			<.001
No		Reference		
Yes		0.17	0.16-0.18	<.001
Unknown		0.53	0.38-0.76	<.001
Radiotherapy	0.277			
No				
Yes				
Chemotherapy	<.001			<.001
No		Reference		
Yes		0.47	0.45-0.48	<.001
Marital status	<.001			<.001
Married		Reference		
Unmarried		1.41	1.37-1.45	<.001
Unknown		1.12	1.05-1.19	0.0312
Insurance situation	<.001			<.001
Insurance		Reference		
No insurance		1.10	1.02-1.20	0.0192
Unknown		0.91	0.82	0.0826
Metastasis	<.001			<.001
None		Reference		
Liver only		3.24	3.11-3.38	<.001
Lung only		2.45	2.22-2.71	<.001
Liver and lung		3.56	3.34-3.80	<.001

RETRACTED

## Data Availability

The data supporting this study's results are available from the corresponding author on request.
